# Can low-carbon pilot policies improve the efficiency of urban carbon emissions?——A quasi-natural experiment based on 282 prefecture-level cities across China

This article has been retracted.

**DOI:** 10.1371/journal.pone.0282109

**Published:** 2023-02-24

**Authors:** Jian Wang, Zhihui Song, Yuzhen Zhang, Rana Yassir Hussain

**Affiliations:** 1 School of Finance and Economics, Jiangsu University, Zhenjiang, Jiangsu, People’s Republic of China; 2 Division of Management and Administrative Sciences, UE Business School, University of Education Lahore, Pakistan; Szechenyi Istvan University: Szechenyi Istvan Egyetem, HUNGARY

## Abstract

Low-carbon pilot policies are an important way to achieve the goal of "peak carbon neutrality" and are of great significance to China’s international commitments. Based on a sample of 282 prefecture-level cities from 2006 to 2020, this paper investigates the impact of low-carbon pilot policies on urban carbon efficiency using a quasi-natural experiment with three batches of low-carbon pilot cities in 2010, 2012, and 2017, respectively. It is found that: (1) low-carbon pilot cities can improve urban carbon emission efficiency, which is still valid after a series of robustness tests such as the parallel trend test, placebo test, PSM-DID, and counterfactual test; (2) low-carbon pilot cities can enhance urban carbon emission efficiency by promoting the level of urban innovation and advanced urban industrial structure; and (3) the impact of low-carbon pilot policies on urban carbon emission efficiency is heterogeneous across cities with different geographical locations, population sizes, and resource endowment types. The findings provide policy insights for the promotion of low-carbon pilot policies and strengthening the construction of low-carbon pilot cities.

## 1. Introduction and literature review

The international community generally believes that carbon dioxide is the main factor causing climate change. The low-carbon development of energy and industry around the world has become the general trend, and carbon emissions have become a global topic of widespread concern. At the climate summit, leaders of all countries made decisions on the determination to cope with climate change, climate adaptability and resilience, climate security, innovative technologies to cope with climate change, and economic opportunities brought about by climate change. China has promised to achieve carbon peak by 2030, that is, carbon dioxide emissions will no longer increase, gradually decrease after reaching the peak, and achieve carbon neutrality by 2060. Achieving the dual-carbon goal is not to stop using energy but to improve carbon emission efficiency by reducing industrial pollution, reducing the use of fossil fuels, increasing energy utilization, and strengthening the use of renewable and clean energy. China is currently in a stage of green and low-carbon development. In 2019, the carbon emission intensity decreased by 48.4% compared with 2005, and the emission reduction effect is remarkable. The report of the 20th National Congress of the Communist Party of China proposed to further promote the energy revolution and strengthen the clean and efficient use of coal, which shows the country’s emphasis on a low-carbon strategy. As the main body of national economic development and social progress, cities undertake most of the social and economic activities and are the main source of national carbon emissions. More than 70% of China ’s carbon emissions come from cities [1], and the improvement of urban carbon emission efficiency is related to the success of the national low-carbon strategy. In order to promote green and low-carbon development and the construction of ecological civilization, since 2010, the Development and Reform Commission has launched three batches of national low-carbon pilot projects, covering 81 cities in 6 provinces, and achieved significant results in reducing urban carbon emissions.

At present, domestic and foreign scholars ’ research on low-carbon pilot and carbon emissions mainly focuses on two aspects. First, the impact of the low-carbon pilot on total factor productivity, ecological efficiency, and the energy environment of enterprises. Such research mostly uses the difference-in-difference method to examine the effectiveness of low-carbon pilot policies. The second is the measurement and influencing factors of regional carbon emission efficiency. This part uses different models to measure carbon emission efficiency, study the time and space evolution of carbon emission efficiency, and study the influencing factors for improving carbon emission efficiency.

For the research on the effect of a low-carbon pilot policy, Emodi, N. V. et al. consider four scenarios through the LEAP model to analyze the impact of different energy policies on the Nigerian energy system. The study discovered that the Nigerian government’s more active policy intervention will result in a reduction in energy demand and greenhouse gas emissions in 2040 [2]; Warbroek, B. investigates the role of LLCEI in the energy transition from the perspective of government governance models and policies supporting local low-carbon energy initiatives [3]; and Chen et al. investigate the win-win path of low-carbon and economy with the policy impact of low-carbon pilot. The study found that low-carbon pilot policies can significantly promote the improvement of total factor productivity in enterprises, and strengthening technological innovation and optimizing resource allocation efficiency are two important transmission mechanisms. This study provides inspiration for the scientific implementation of low-carbon pilot policies [4]; Cheng et al. used the difference-in-difference model to examine the impact of China’s low-carbon pilot policy on urban green GDP at the prefecture-level city level and found that low-carbon city construction has a scale effect and regional differences [5]; Gehrsitz, M. used the difference-in-difference method to explore the impact of low-emission areas on air pollution. He found that Germany’s low-carbon regional policy can reduce local pollution levels [6]; Tang et al. evaluated the effect of China’s low-carbon pilot by the difference-in-difference method. The results show that the low-carbon pilot policy has played a role in the land transfer of energy-intensive industries to a certain extent, but the policy effect gradually weakened over time [7]; Zhou et al. used the low-carbon pilot policy as an example to explore the impact of environmental regulation policies on corporate energy-saving behavior. The study found that the low-carbon pilot policy significantly reduced corporate coal consumption and coal intensity, and this policy is heterogeneous, which is manifested in the fact that energy-intensive industries and state-owned enterprises bear more energy-saving tasks [8]. In order to overcome endogenous problems, economists often use a variety of econometric tools to estimate the treatment effect of policies by means of "quasi-experiment" opportunities. Common methods include the instrumental variable method, regression discontinuity design, propensity score matching method, and double difference method; each of these methods has its own advantages and disadvantages [9]. This paper focuses on the DID method, which is popular with policy evaluators because of its rapid development. The DID method was introduced into the field of economic research in the West as early as the late 1970s [10]. The earliest authoritative literature on the introduction of the DID method in China was Zhou and Chen’s research on the impact of tax reform on farmers’ income growth [11]. Because of the many advantages of the DID method, it has been widely used in medical, e-commerce, finance, agriculture, and other aspects. Schreyögg J. and Grabka MM use the difference-in-difference method to explore the impact of German outpatient care co-payments on the overall needs of doctors [12]; Wang et al. found that e-commerce can significantly reduce agricultural non-point source pollution [13]; Kim et al. explored whether the expansion of dental insurance for the elderly would have an impact on dental care needs [14]; and Adam et al. found that even after the adoption of the farmer empowerment method, the problems of agricultural production factors and rice yield in Indonesia still exist [15].

In terms of the measurement and influencing factors of regional carbon emission efficiency, Zhao et al. used the DEA model to measure the carbon emission efficiency of the transportation sector in 30 provinces of China from 2010 to 2016 and explored its influencing factors through the spatial Dubin model. The study found that technological progress is a key factor in improving the carbon emission efficiency of the transportation sector and that the increase in the share of waterway and railway transportation modes contributes to the improvement of transportation carbon emission efficiency [16]; Wang et al. used data envelopment analysis (DEA) to measure carbon emission efficiency and carbon emission technology gap ratio at the provincial level in China, and found that carbon emission efficiency in various regions of China is heterogeneous [17]; Wang et al. used the GMM method to analyze the panel data of 131 countries to explore the impact of industrialization and renewable energy on carbon emission efficiency and analyze the mode of action and interaction of influencing factors. The study found that there was heterogeneity in the factors affecting carbon emission efficiency in high-income and low-income countries, and the rise of renewable energy and industrialization improved carbon emission efficiency [18]; Quan et al. used the IPCC method to calculate the total carbon emissions of China’s logistics industry and used the LMDI decomposition model to decompose the influencing factors of carbon emissions into five aspects, explore the mechanism of each factor on carbon emissions, and put forward reasonable policy recommendations [19].

In summary, the existing literature has conducted in-depth research on low-carbon pilot and carbon emission efficiency from different perspectives, but there are still the following limitations: (1) Most scholars discuss low-carbon pilot policies and carbon emission efficiency separately and rarely explore the internal relationship between low-carbon pilot policies and urban carbon emission efficiency; (2) Although the existing literature has done a lot of research on environmental regulation and technological innovation, that is, to verify the "Porter hypothesis," most of the existing literature has a single means of implementing environmental policies, and the research on the comprehensive environmental policy of low-carbon pilot is still in its infancy.

By analyzing the shortcomings of the existing literature, this paper focuses on the effect and mechanism of a low-carbon pilot policy on carbon emissions, measures it through the difference-in-difference model, and analyzes the mediating effect and heterogeneity. The contributions of this paper are: (1) To broaden the topic of environmental policy, analyze the policy effect of the low-carbon pilot, which is a comprehensive environmental policy, and enrich the content of the "Porter hypothesis." (2) Based on the undesirable output SBM model to measure the urban carbon emission efficiency, using the DID model to test the impact mechanism of a low-carbon pilot policy on urban carbon emission efficiency, and through a series of robustness tests to verify the validity of the results; (3) From the perspectives of innovation level and industrial upgrading, this paper discusses the internal influence mechanism of a low-carbon pilot policy on urban carbon emission efficiency and the heterogeneity of different types of cities.

## 2. Theoretical analysis and research hypothesis

As the main body of China ’s society and economy, cities bear most of the social and economic activities. Most of China’s carbon emissions come from cities. Reducing urban carbon emissions and improving urban carbon emission efficiency are inevitable requirements of sustainable development. Therefore, in the context of the country’s emphasis on carbon emission constraints, cities pay more attention to green and low-carbon sustainable development and the effective improvement of carbon emission efficiency [20]. The implementation of low-carbon pilot policies can effectively accelerate the transformation of cities toward innovative level development, reasonable industrial structure, efficient energy utilization, and carbon emission efficiency improvement.

The impact of environmental regulation has always been controversial: some scholars believe that environmental regulation has " innovation compensation effect " according to the " Porter hypothesis, " [21] that is, reasonable environmental regulation will promote enterprises to carry out technological innovation and environmental protection technology upgrading [22,23], thereby improving urban carbon emission efficiency; According to the "follow the cost effect," [24] some scholars believe that environmental regulation will increase costs, crowd out urban production and R&D investment space [25], and then slow down the growth rate of urban carbon emission efficiency. The low-carbon pilot policy is a comprehensive environmental regulation policy at the city level. Improving the carbon emission efficiency of cities to achieve a win-win situation between carbon emission reduction and economic development is the primary goal of pilot city construction. Many studies have confirmed that low-carbon pilot policies can effectively reduce urban carbon emissions [26,27]. Based on this, this paper proposes the following hypothesis:

**Hypothesis H1: Low-carbon pilot policies have significantly improved urban carbon emission efficiency.**

Grossman et al. proposed the decomposition of the environmental effects of economic growth, and the impact of various factors on the environment can be summarized as scale effect, structural effect, and technical effect. The level of innovation and the upgrading of industrial structure are the main driving forces for the sustainable development of regional economy [28]. Considering that the main goal of low-carbon pilot city construction is a win-win situation of carbon emission reduction and economic construction, this paper argues that low-carbon pilot policies can promote urban carbon emission efficiency by improving urban innovation levels and industrial structure upgrading. The reasons are as follows:

On the one hand, the low-carbon pilot policy advocates for local governments to cultivate a low-carbon industrial system, focus on the development of new industries and modern services, and pay more attention to the development of the tertiary industry [29]; on the other hand, the low-carbon pilot policy promotes the relocation of high-pollution and high-emission industries, raises barriers to entry for high-pollution and high-emission industries, and effectively promotes cities to move towards advanced industrial structures [30], which in turn verifies the "pollution paradise" hypothesis. At the same time, after the implementation of the low-carbon pilot policy, the state advocates a green and sustainable lifestyle, consumers’ awareness of environmental protection is improved, they will be more inclined to buy green environmental protection products, demand promotes supply, and the benefits of green low-carbon industries and public demand will gradually expand the market size [31]. The demand of most consumers and the expansion of market scale will attract more investment and promote the upgrading of industrial structures [32].

Most low-carbon pilot cities emphasize technological innovation as the driving force for the development of low-carbon industries [33]. Therefore, cities can upgrade their processes by increasing technological research and innovation, relying on technological advances in production and low-carbon environmental technologies to reduce carbon emissions and compensate for the loss of environmental costs [34], thus improving carbon efficiency. In addition, the low-carbon pilot policy requires cities to reduce emissions and pollution, and environmental constraints force cities to undertake autonomous technological innovation to reduce the cost of green production, thus validating the "innovation compensation effect." Accordingly, this paper proposes the following hypothesis:

**Hypothesis H2a: Low-carbon pilot policies improve urban carbon efficiency by promoting advanced industrial structures.**
**Hypothesis H2b: Low-carbon pilot cities improve urban carbon efficiency by promoting innovation levels.**

China ’s vast territory, all low-carbon pilot cities will be subject to low-carbon policy regulation, but because of the size of the city, resource endowment, environmental awareness, the level of economic development are very different, resulting in different urban carbon emissions costs and environmental compliance costs are very different, and different levels of development in various regions led to different levels of technology and awareness of the masses, so that different regions of the policy regulation and attention to different ways. Many studies have confirmed that the low-carbon pilot policy has had a heterogeneous impact on total factor productivity [35], corporate green innovation technology [36] and urban carbon emissions [37] in different regions. Accordingly, this paper proposes the following hypothesis:

**Hypothesis H3: There is heterogeneity in the impact of low-carbon pilot policies on carbon emission efficiency.**

## 3. Study design and data description

### 3.1 Model construction

#### 3.1.1 Super-efficient SBM models that include non-desired outputs

The SBM model is a non-radial, non-angular DEA model that can solve the slackness problem by adding non-desired output variables and correcting for slack variables, but it produces multiple efficiency values of 1, making it difficult to compare decision units [38]. Tone combines super-efficient DEA with SBM to remove the super-efficient SBM model, which allows for the continued decomposition of units with efficiency values of 1. improves the applicability of the model [39,40]. In this paper, based on the input-output perspective, the over-efficient SBM model is applied to measure the carbon emission efficiency of 282 prefecture-level cities in China from 2006 to 2020, and the model is set as follows:

$$min\rho =\frac{1+\frac{1}{M}\sum_{i=1}^{M}\frac{\omega_{i}^{-}}{x_{ik}}}{1-\frac{1}{U_{1}+U_{2}}(\sum_{s=1}^{U_{1}}\frac{\omega_{s}^{d}}{y_{sk}^{d}}+\sum_{q=1}^{U_{2}}\frac{\omega_{q}^{t}}{y_{qk}^{t}})}$$

$$s.t.\left\{ \begin{array}{c} x_{ik}\geq \sum_{j=1,j\neq k}^{n}x_{ij}\lambda_{j}+\omega_{i}^{-}\\ y_{sk}^{d}\geq \sum_{j=1,j\neq k}^{n}x_{sj}^{d}\lambda_{j}-\omega_{s}^{d}\\ y_{qk}^{t}\geq \sum_{j=1,j\neq k}^{n}x_{qj}^{t}\lambda_{j}+\omega_{q}^{t}\\ \lambda_{j}\geq 0,j=1,2,\cdots n\\ \omega_{i}^{-}\geq 0,i=1,2,\cdots M\\ \omega_{s}^{d}\geq 0,s=1,2,\cdots U_{1} \end{array}\right.$$ (1)

Where it is assumed that there are *n* DMU, each DMU consists of M input elements, *U*_1_ desired output elements and *U*_2_ non-desired output elements, *ρ* is the measured DMU efficiency value, *λ*_*j*_ is the weight vector of the DMU, $x_{ik}、y_{sk}^{d}、y_{qk}^{t}$ are the input matrix elements, desired output matrix elements and non-desired output matrix elements respectively, $\omega_{i}^{-}、\omega_{s}^{d}、\omega_{q}^{t}$ are input element slack, desired output element slack and non-desired output element slack. The DMU is valid when *ρ*≥1; when *ρ*<1,the DMU is invalid.

#### 3.1.2 Multi-period DID model

Traditional DID assumes that all individuals in the treatment group start to receive policy shocks at exactly the same point in time, but there will be inconsistencies in the point in time when individuals in the treatment group receive treatment. The low carbon pilot policy explored in this paper was opened in three batches in 2010, 2012, and 2017, respectively, and traditional DID can no longer satisfy, so this paper refers to relevant literature [41], cites studies by Beck et al. [42,43] and constructs a multi-period DID model, which is set as follows:

$${DEE}_{i,t}=\beta_{0}+\beta_{1}{TREAT}_{i}\times {POST}_{t}+\rho X_{i,t}+\mu_{i}+\gamma_{t}+\varepsilon_{i,t}$$ (2)

Where *DEE*_*i*,*t*_ is the carbon emission efficiency of city i in year t; *TREAT*_*i*_×*POST*_*t*_ is a dummy variable, which takes 1 if city i is a low-carbon pilot city and is after the implementation of the low-carbon pilot policy, otherwise it takes 0; *X*_*i*,*t*_ is a control variable; *μ*_*i*_ and *γ*_*t*_ denote city fixed effects and time fixed effects respectively; *ε*_*i*,*t*_ is a random error term.

### 3.2 Variable setting

#### 3.2.1 Explained variable

The explained variable is carbon emission efficiency, and this paper adopts the super-efficient SBM model to measure urban carbon emission efficiency from the input-output perspective. The system of measurement indicators is shown in Table 1. The capital factor is represented by fixed capital stock, measured by the perpetual inventory method of Zhang [44], and deflated using 2006 as the base period; the labor factor and energy factor are represented by year-end unit employees and total annual electricity consumption, respectively; the desired output is represented by real GDP, calculated using the GDP deflator using 2006 as the base period; and the non-desired output is represented by carbon dioxide emissions.

**Table 1:** Carbon efficiency input-output indicator system.

Target level	Guideline level	Indicator layer	Unit	Indicator meaning
Carbon efficiency	Input indicators	Fixed capital stock	billion	Capital elements
		Number of employees in the unit at the end of the year	million people	Labor elements
		Total annual electricity consumption	million kWh	Energy elements
	Output indicators	Real GDP	billion	Desired output
		CO2 emissions	billion tons	Non-desired outputs

#### 3.2.2 Core explanatory variables

The core explanatory variable in this paper is the dummy variable *TREAT*_*i*_×*POST*_*t*_, which is 1 if city *i* is a low carbon pilot city and is after the implementation of the low carbon pilot policy and 0 if city *i* is not a low carbon pilot city or city *i* is a low carbon pilot city but is before the implementation of the low carbon pilot policy. It is worth noting that the second batch of pilot cities was established in December 2012, so this paper chooses 2013 as the policy shock point and uses the 2012 policy shock as a robustness test.

#### 3.2.3 Control variables

The following control variables are used in this paper: (1) GDP per capita (PGDP), expressed as the ratio of real gross product to population in cities; (2) population density (PD), expressed as the ratio of the number of people in a city to its administrative area; (3) R&D investment (RD), expressed as the ratio of research expenditure to fiscal expenditure; (4) foreign investment intensity (FDI), expressed as the ratio of actual foreign investment used to GDP; (5) educational attainment (EDU), expressed in terms of the number of students enrolled in higher education.

#### 3.2.4 Mediating variables

The following mediating variables are used in this paper: (1) innovation level (ino), expressed as the number of patents granted; (2) the index of industrial structure upgrading (isad), which is obtained by referring to the practice of Yuan and Zhu through the proportion of the output value of the first, second, and third industries in GDP [45].

### 3.3 Data sources

In order to ensure the availability and accuracy of data, this paper selects 282 prefecture-level cities in China from 2006 to 2020 for research. All data are derived from the "China Urban Statistical Yearbook," "China Energy Statistical Yearbook," and other statistical yearbooks and statistical bulletins of various provinces and cities. The missing data are filled by the linear interpolation method and the trend prediction method. The descriptive statistics of the data are shown in Table 2 below. Heterogeneity analysis of regional division comes from the National Bureau of Statistics China is divided into three regions: the eastern region, including Beijing and other 11 provinces (cities); the central region includes 8 provinces such as Shanxi; the western region includes 12 provinces including Shaanxi. The division of urban scale is derived from the "Notice of the State Council on Adjusting the Criteria for the Division of Urban Scale." Based on the permanent population of municipal districts in 2015, cities with a population of more than 1 million are large cities; cities with a population of 500000 to 1 million are medium-sized cities; and cities with a population of less than 500,000 are small cities. Resource endowment division comes from the State Council’s "national resource-based city sustainable development plan."

**Table 2:** Results of descriptive statistics for variables.

Variables	N	Mean	Std. Dev.	Min	Max
*DEE*_*i*,*t*_	4,230	0.587487	0.0680034	0.4316439	0.9012441
*PGDP*	4,230	44209.22	32924.83	2767	467749
*PD*	4,230	453.3083	420.3577	4.7	4262.103
*RD*	4,230	1.485893	1.540031	0.0270804	20.68348
*FDI*	4,230	0.0265415	0.3438716	4.8979e-07	22.33837
*EDU*	4,230	87926.3	159562.1	231	1307144
*ino*	4,230	4470.381	12349.29	0	222412
*isad*	4,230	2.26949	0.14525	1.831	2.8357

## 4. Empirical results and analysis

### 4.1 Time-series evolutionary characteristics of carbon emission efficiency

In order to analyze the time-series evolution of carbon emission efficiency, this paper uses the kernel density estimation method to portray the time-series trend evolution of carbon emission efficiency in China (Fig 1). As shown in the figure, the distribution pattern of carbon emission efficiency in China shows the following characteristics: First, the center of the kernel density distribution curve tends to move to the right with increasing years, indicating an upward trend in overall carbon emission efficiency; second, the width of the main peak narrows over time, indicating that the gap in carbon emission efficiency among cities becomes smaller; third, the number of peaks did not show a double-peak phenomenon, indicating that China’s carbon emission efficiency has no polarization phenomenon.

**Fig 1:** Kernel density estimates of the time-series evolution of carbon emissions efficiency.

### 4.2 Baseline regression

Table 3 reports the baseline regression results of the impact of low-carbon pilot policies on urban carbon emission efficiency. Model (1) represents the benchmark regression results without control variables and individual time fixed effects. Model (2) adds individual time-double fixed effects on the basis of Model (1). Model (3) shows the regression results of an unfixed individual time-fixed effect while adding control variables such as per capita GDP, population density, R&D investment, foreign investment intensity, and education level. Model (4) shows the benchmark regression results of adding control variables while adding individual time factors. It can be seen from the table that no matter whether the fixed effect is controlled or the control variables are added, the estimated coefficient of carbon emission efficiency of the low-carbon pilot policy cities is significantly positive at the level of 1%, which indicates that the low-carbon pilot policy significantly improves the urban carbon emission efficiency and verifies the correctness of Hypothesis H1.

**Table 3:** Impact of low-carbon pilot policies on the efficiency of urban carbon emissions.

Variables	Model (1)	Model (2)	Model (3)	Model (4)
	*DEE*_*i*,*t*_	*DEE*_*i*,*t*_	*DEE*_*i*,*t*_	*DEE*_*i*,*t*_
TREAT×POST	0.0368*** (0.00374)	0.00889*** (0.00298)	0.0327*** (0.003828)	0.00915*** (0.00305)
*PGDP*			6.01e-07*** (3.93e-08)	9.78e-08* (5.24e-08)
*PD*			-2.32e-06 (2.81e-06)	-7.86e-06** (3.80e-06)
*RD*			-0.00499*** (0.000873)	0.00155** (0.000755)
*FDI*			-0.000984 (0.00291)	-0.000286 (0.00177)
*EDU*			-7.43e-08*** (7.22e-09)	1.13e-09 (1.92e-08)
Constant	0.584*** (0.00108)	0.5161*** (0.01019)	0.5732*** (0.00181)	0.545*** (0.00295)
City FE	NO	YES	NO	YES
Year FE	NO	YES	NO	YES
N	4230	4230	4230	4230
R^2^	0.0224	0.7069	0.0875	0.7085

Note: The standard error of clustering to the city level is indicated in parentheses. * * *, * *, and * are significant at 1%, 5% and 10% levels, respectively.

In terms of control variables, it can be seen from the benchmark regression results of Model 4 that the estimated coefficient of the impact of per capita GDP (PGDP) on urban carbon emission efficiency is 9.78e-08 and passes the 10% significance test, which indicates that the increase in per capita GDP can promote the efficient transformation of carbon emission efficiency. Regions with a higher level of economic development will carry out the transformation and upgrading of the industrial structure earlier because the industrial structure is relatively perfect and the government has higher requirements and more economic input for regional management and pollution prevention, which will promote the improvement of carbon emission efficiency. The estimated coefficient of population density (PD) is -7.86e-06, which is significantly negative at the 5% level. The increase in population will lead to a large concentration of human activities, promote energy consumption, further increase carbon emissions, and thus reduce carbon emission efficiency. The estimated coefficient of R&D investment (RD) is 0.00155, which is significantly positive at the 5% level. This shows that the higher the R&D investment, the higher the carbon emission efficiency will be. In regions with higher R&D investment, the government and the public pay more attention to innovation and development. The attention of the masses is the fundamental driving force for the improvement of the innovation level, so R&D investment is significantly positively correlated with carbon emission efficiency. The intensity of foreign capital (FDI) is negatively correlated with carbon emission efficiency, but not significantly, which further verifies the "pollution haven" hypothesis; education (EDU) has no significant effect on carbon emission efficiency.

### 4.3 Robustness tests

#### 4.3.1 Parallel trend test

The above benchmark regression shows that low-carbon policy pilots can improve urban carbon emission efficiency, but it cannot be ruled out that this result existed before the implementation of the policy. Therefore, it is necessary to pass the “parallel trend test,” that is, to test that there is no significant difference in carbon emission efficiency among cities, before the implementation of the policy. In this paper, we take the time trend of non-low carbon pilot cities and low carbon pilot cities in the 7 periods before and after the policy implementation, using 2013 as the base period, and plot the parallel trend test. As shown in Fig 2, when *k*<0, i.e., the 95% confidence interval before the implementation of the policy, contains 0, i.e., *β*_*k*_ is not significantly different from 0, which indicates that there is no significant difference between the carbon emission efficiency of low-carbon pilot cities and non-low-carbon pilot cities before the implementation of the low-carbon pilot policy. When *k*≥0, *β*_*k*_ is all significantly positive and generally tends to increase, indicating that the low-carbon pilot policy has indeed effectively improved the carbon emission efficiency of cities.

**Fig 2:** Parallel trend test.

#### 4.3.2 Placebo test

Considering that urban carbon emission efficiency may also be subject to shocks from other variables, and in order to rule out the possibility of low carbon pilot policies acting in conjunction with other stochastic factors, this paper uses a placebo approach to test the robustness of the model regression results. The same number of cities as the low-carbon pilot cities were randomly selected as the experimental group, and the other cities were used as the control group to construct dummy variables for regression. In this paper, 500 and 1000 randomized trials were conducted, and 500 and 1000 estimated coefficients were generated, as shown in Figs 3 and 4, respectively. From the graph, it can be seen that whether there are 500 or 1000 random tests, the estimation coefficients of low-carbon pilot policies on urban carbon emission efficiency are mostly concentrated near the zero point and obey the normal distribution. The p values of most estimates are greater than 0.1 (the horizontal dotted line in the graph), that is, they are not significant at the 10% level, which indicates that the impact of low-carbon pilot policies on carbon emission efficiency is not accidental and is not affected by other random factors, further verifying the robustness of the benchmark regression.

**Fig 3:** 500 estimate placebo test.

**Fig 4:** 1000 estimate placebo test.

#### 4.3.3 Other robustness tests

The above study found that low-carbon pilot policies can significantly improve the efficiency of urban carbon emissions. To verify the reliability of the previous findings, this paper also employs the following robustness tests:

1. **Estimation based on the PSM-DID method**
  The use of the DID method requires meeting the assumption that the experimental group has the same trend as the control group. To circumvent the endogeneity problem caused by selectivity bias, this paper uses the PSM-DID method to test the impact of low-carbon pilot policies on the efficiency of urban carbon emissions. Logit regression was performed with the control variables as covariates to calculate propensity matching scores. Then DID estimation was performed using the K-nearest neighbor matching method for the successfully matched samples and the samples satisfying the common support assumptions, respectively, and the results are shown in columns (1) and (2) of Table 4. The table shows that the impact of the low carbon pilot policy on carbon emissions is positively significant at the 1% level for both the matched successful sample and the sample meeting the common support assumption, proving that the baseline regression results are robust.
2. **1% top and bottom indent processing on a continuous basis**
  The continuous variables required for this paper were all subjected to the upper and lower 1% tailing process, followed by the estimation of the model, and the results are shown in column (3). As can be seen from the table, the impact of low-carbon pilot policies on carbon emissions is positively significant at the 10% level, proving the robustness of the baseline regression results.
3. **Exclusion of municipalities directly under the Central Government**
  Considering that municipalities directly under the central government have greater specificity in terms of policy support and economic development level at the national level, this paper excludes municipalities directly under the central government for difference-in-difference estimation, and the results are shown in column (4), where the effect of low carbon pilot policies on carbon emission efficiency is significantly positive at the 5% level, verifying the robustness of the previous results.
4. **Counterfactual test**
  In order to avoid the regression bias caused by possible missing variables, this paper adopts the counterfactual test method to verify the robustness, i.e., the policy implementation time is advanced by 1 year and 2 years, respectively, and the difference-in-difference estimation is carried out. The results are shown in columns (5) and (6). It is known from the table that the impact of low-carbon pilot policies on carbon emission efficiency has not passed the significance test, which proves the reliability of the previous results.

**Table 4:** Other robustness tests.

	PSM-DID		Data trailing 1%	Excluding municipalities	Counterfactual test	
	Sample Matching Success	Meeting the common support assumptions			Policy point in time 2012	Policy point in time 2011
	(1)	(2)	(3)	(4)	(5)	(6)
	*DEE*_*i*,*t*_	*DEE*_*i*,*t*_	*DEE*_*i*,*t*_	*DEE*_*i*,*t*_	*DEE*_*i*,*t*_	*DEE*_*i*,*t*_
TREAT×POST	0.04698*** (0.00855)	0.04281*** (0.00716)	0.00368* (0.00207)	0.00951** (0.00312)	0.00891 (0.00603)	0.0896 (0.00605)
Control variables	YES	YES	YES	YES	YES	YES
Constant	0.5825*** (0.00722)	0.5804*** (0.00537)	0.54083*** (0.00243)	0.54660*** (0.00298)	0.54522*** (0.00357)	0.54515*** (0.00358)
City FE	YES	YES	YES	YES	YES	YES
Year FE	YES	YES	YES	YES	YES	YES
N	1298	4182	4230	4158	4230	4230
R^2^	0.1532	0.1112	0.7776	0.3811	0.3867	0.3867

## 5. Analysis of impact mechanisms

The above studies show that low-carbon pilot policies can significantly improve urban carbon emission efficiency, but their impact mechanism needs specific analysis. Based on the above analysis and existing studies, this paper studies the specific path of the impact of low carbon pilot policies on carbon emission efficiency from the perspectives of innovation level and advanced industrial structure, drawing on the studies of Baron and Kenny [46] and Li and Zou [47] to construct a mediating effect model through Eqs (3) and (4).

$$M_{it}=\alpha_{0}+\beta Treat_{i}\times post_{t}+\delta X_{it}+\vartheta_{t}+\mu_{i}+\varepsilon_{it}$$ (3)

$${CEE}_{it}=\alpha_{0}+\beta Treat_{i}\times post_{t}+\theta M_{it}+\delta X_{it}+\vartheta_{t}+\mu_{i}+\varepsilon_{it}$$ (4)

Where *M*_*it*_ represents the mediating variable, this paper uses the innovation level expressed by the number of patents granted and the index of advanced industrial structure calculated by the proportion of primary, secondary, and tertiary industries in GDP, and the formula is shown in Eq (5), where *y*_*m*_ represents the proportion of the output value of industry m in GDP.


$$isad=\sum_{m=1}^{3}y_{m}\times m$$ (5)

Table 5 reports the results of the stepwise regression method used to test the mediating mechanism. The coefficient of the dummy variable in column (1) is significantly positive at the 1% level, indicating that low-carbon pilot policies can significantly contribute to the improvement of the level of innovation; the coefficients of the dummy variable and the level of innovation in column (2) are both significant at the 1% level, which leads to the conclusion that low-carbon pilot policies can improve the efficiency of urban carbon emissions by promoting the progress of the level of innovation, proving the accuracy of hypothesis H2a. The coefficient of the dummy variable in column (3) is significantly positive at the 1% level, indicating that the implementation of low carbon pilot policies can accelerate the transformation of industrial structure to advanced; the coefficients of the dummy variable and advanced industrial structure in column (2) are both significant at the 1% level, thus it can be concluded that low carbon pilot policies can improve the efficiency of urban carbon emissions by promoting advanced industrial structure, supporting hypothesis H2b.

**Table 5:** Analysis of intermediary mechanisms.

	(1)	(2)	(3)	(4)
Variables	*ino*	*DEE*_*i*,*t*_	*isad*	*DEE*_*i*,*t*_
TREAT×POST	0.326078*** (0.056354)	0.022972*** (0.003222)	0.039983*** (0.004569)	0.21521*** (0.0032587)
*ino*		0.014173*** (0.000879)		
*isad*				0.154674*** (0.10766)
Control variables	YES	YES	YES	YES
Constant	4.949897*** (0.0606115)	0.476121*** (0.0056189)	2.16592*** (0.005900)	0.212008*** (0.023554)
N	4230	4230	4230	4230
R^2^	0.5247	0.2665	0.3756	0.2639

In order to verify the robustness of the results obtained, the Sobel test and the Bootstrap test were used to test the results. The p-values for the Sobel test were less than 0.05, and the confidence intervals for the Bootstrap test did not contain 0. The original hypothesis was rejected, and the robustness of the mediation mechanism test was verified.

## 6. Heterogeneity analysis

The above study examines the impact of low-carbon pilots on carbon emission efficiency based on the overall level of 282 prefecture-level cities in China. However, China has a vast territory, and only starting from the overall situation may cover regional differences caused by different city sizes, resource endowments, environmental awareness, and economic development levels. In view of this, this paper further explores whether there is heterogeneity in the impact of low-carbon pilot policies on carbon emissions. Specifically, China’s cities are divided into eastern cities, central cities, and western cities according to geographical location [48]; according to the "Notice of the State Council on Adjusting the Standards for Dividing City Size," cities are divided into large cities, medium-sized cities, and small cities according to the number of permanent residents [49]; cities shall be divided into resource-based cities and non-resource-based cities according to the requirements of the “National Sustainable Development Plan for Resource-based Cities" of the State Council [50].

### 6.1 Examining regional heterogeneity

Table 6 reports the results of the heterogeneity analysis of the impact of low-carbon pilot cities on carbon emission efficiency in the eastern, central, and western regions. It can be seen from the table that the impact of low-carbon pilots on carbon emission efficiency in the eastern and western regions is significantly positive at the 5% level, which verifies the significant promotion effect of low-carbon pilots on carbon emission efficiency. The central low-carbon pilot effect is not significant. The eastern cities have significant advantages in urban economic development level, high-tech, personnel training, and education, which can provide good policy and economic support for improving carbon emission efficiency and further verify the “Porter hypothesis “; after the in-depth implementation of the national “western development” strategy, the western region has received national support policies, and the economic foundation, ecological environment, and industrial structure have been greatly improved, thus promoting the improvement of carbon emission efficiency; due to the "rise of central China" strategic policy, the central region is in a period of tackling difficulties and creating a new situation with the rise of central China. It may be due to the development of high-energy-consuming industries in the region, increasing the difficulty of carbon emission reduction work and resulting in a low-carbon pilot policy on carbon emission efficiency that is not significant.

**Table 6:** Examining regional heterogeneity.

Variables	Eastern	Central	Western
	*DEE*_*i*,*t*_	*DEE*_*i*,*t*_	*DEE*_*i*,*t*_
TREAT×POST	0.00576** (0.00249)	-0.00192 (0.00168)	0.01684** (0.007382)
Control variables	YES	YES	YES
Constant	0.5436*** (0.00207)	0.29328*** (0.003968)	0.3764*** (0.01215)
City FE	YES	YES	YES
Year FE	YES	YES	YES
N	1500	1485	1245
R^2^	0.6908	0.9288	0.4231

### 6.2 Examining city-size heterogeneity

Table 7 reports the heterogeneity of the impact of low-carbon pilot policies on carbon emission efficiency in terms of city size. As can be seen from the table, the impact of low-carbon pilots in large cities on carbon emission efficiency is significantly positive at the 5% level; while low-carbon pilot policies in medium and small cities have no significant effect on carbon emission efficiency, indicating that the impact of low-carbon pilot policies on carbon emission efficiency is obvious in large cities but not obvious in small and medium-sized cities. It may be due to the good economic foundation and human resources of big cities, which can attract the inflow of talents, form industrial agglomerations and factor agglomerations, attach importance to sustainable development strategies, and give full play to the positive driving effect of a low-carbon pilot policy on carbon emission efficiency.

**Table 7:** Examining city-size heterogeneity.

Variables	Big Cities	Medium Cities	Small Cities
	*DEE*_*i*,*t*_	*DEE*_*i*,*t*_	*DEE*_*i*,*t*_
TREAT×POST	0.0028129** (0.001222)	-0.0029964 (0.004405)	0.0155841 (0.0108138)
Control variables	YES	YES	YES
Constant	0.332446*** (0.0036298)	0.353297*** (0.0081165)	0.361770*** (0.016675)
City FE	YES	YES	YES
Year FE	YES	YES	YES
N	2160	1365	705
R^2^	0.9020	0.6581	0.4637

### 6.3 Examining the heterogeneity of urban resource endowments

Table 8 reports the heterogeneity of the impact of low-carbon pilot policies on carbon emission efficiency in cities with different resource endowments. It can be seen from the table that the low-carbon pilot policy of resource-based cities has a significant positive impact on urban carbon emission efficiency at the 1% level, while the low-carbon pilot policy of non-resource-based cities has no significant impact on urban carbon emission efficiency. The reason may be that the industry and other resource-based industries in resource-based cities are relatively more developed, have a higher degree of dependence on energy, and are more likely to form “path dependence.” Some resource-based cities are still in the stage of undertaking high pollution and high energy consumption areas, facing the challenge of urban transformation. After the implementation of the low-carbon pilot policy, government regulation has promoted the green transformation of cities to a certain extent, improved the long-term and efficient mechanisms of sustainable development, advocated the development of low-carbon industries, reduced carbon emissions, and thus improved carbon emission efficiency. Non-resource-based cities are less dependent on energy and are less regulated by national low-carbon pilot policies. Therefore, the impact of low-carbon pilot policies on non-resource-based cities’ carbon emission efficiency is not significant.

**Table 8:** Examining the heterogeneity of urban resource endowments.

Variables	Resource-based	Non-resource based
	*DEE*_*i*,*t*_	*DEE*_*i*,*t*_
TREAT×POST	0.02052*** (0.00494)	0.00072 (0.00249)
Control variables	YES	YES
Constant	0.32018*** (0.00579)	0.38814*** (0.00784)
City FE	YES	YES
Year FE	YES	YES
N	1705	2513
R^2^	0.6788	0.6059

In summary, the previous hypothesis H3 holds.

## 7.Test for spatial spillover effect

According to the above analysis, the implementation of a low-carbon pilot policy can promote the improvement of urban carbon emission efficiency, and its impact on urban carbon emission efficiency has regional heterogeneity. This paper further verifies whether the spatial spillover effect between regions will affect the relationship between the low-carbon pilot policy and urban carbon emission efficiency.

Table 9 shows that whether an economic distance matrix, an economic geography nested matrix, or an inverse distance matrix is introduced, the coefficient of the impact of low-carbon pilot policies on urban carbon emission efficiency is positive and all passed the 1% significance test, indicating that it has significant spatial effects, that is, local implementation of low-carbon pilot policies will also significantly promote the improvement. At the same time, the spatial term coefficient ρ of the model is significantly positive at the 1% level, and the interaction term W×TREAT×POST coefficient is significantly positive when the economic distance matrix and the inverse distance matrix are introduced, indicating that each region not only has an exogenous low-carbon pilot policy interaction effect in space but also has an endogenous interaction effect on urban carbon emission efficiency. In view of the simple point regression results used to analyze the spatial spillover effect between regions, the regression coefficient value of the spatial interaction term cannot be directly used to discuss the marginal impact of the implementation of low-carbon pilot policies on urban carbon emission efficiency. Therefore, it is necessary to use direct and indirect effects to explain the impact of core explanatory variables in a region on the explained variables in the region and other regions. The results are shown in Table 9. It can be seen that the indirect effect of low-carbon pilot policies on urban carbon emission efficiency is significant.

**Table 9:** Spatial econometric model regression results.

	Economic distance matrix	Economic geography nested matrix	Anti-distance matrix	
			equation of the first degree	square
TREAT×POST	0.01331*** (0.00307)	0.00957*** (0.00297)	0.01016*** (0.00296)	0.01231*** (0.00297)
W×TREAT×POST	0.07464*** ((0.00708)	0.01616 (0.01133)	0.03763*** (0.01293)	0.04181*** (0.00973)
Ρ	0.44065*** (0.02254)	0.82517*** (0.03418)	0.84883*** (0.03105)	0.66042*** (0.02487)
Control variables	YES	YES	YES	YES
City FE	YES	YES	YES	YES
Year FE	YES	YES	YES	YES
Direct effect	0.01866*** (0.00313)	0.01007*** (0.00298)	0.01128*** (0.00299)	0.01478*** (0.00299)
Indirect effect	0.13750*** (0.01123)	0.13149*** (0.04483)	0.30409*** (0.06584)	0.14239*** (0.02292)
N	4230	4230	4230	4230
R^2^	0.2914	0.3377	0.3342	0.3155

## 8. Conclusions and recommendations

Low-carbon pilot policies can effectively promote the improvement of urban carbon emission efficiency. Using panel data from 282 prefecture-level cities across China from 2006 to 2020 as a sample, this paper examines the impact of low-carbon pilot policies on urban carbon emission efficiency using a difference-in-difference method and finds that low-carbon pilot policies have a significant positive effect on urban carbon emission efficiency. This conclusion is still valid after robustness tests such as the parallel trend test, placebo test, PSM-DID test, data down the tail of 1%, excluding municipalities, and the counterfactual test. Mechanism analysis shows that a low-carbon pilot policy will promote carbon emission efficiency by improving the level of urban innovation and industrial structure upgrades. The impact of low-carbon pilot policies on carbon emission efficiency is heterogeneous in cities of different regions, cities of different sizes, and cities with different resource endowments. Further research finds that there is a spatial spillover effect on the impact of low-carbon pilot policies on urban carbon emissions.

The conclusions of this paper provide the following policy insights for effectively improving the efficiency of urban carbon emissions:

1. The low-carbon pilot policy has been effective in promoting urban carbon efficiency, confirming the sound decision to implement the government’s low-carbon pilot policy. Therefore, while strengthening the construction of low-carbon pilot cities, the implementation of low-carbon pilot policies should be vigorously promoted, and more cities should be gradually included in the scope of the pilots. For cities with good demonstration effects or significant achievements, policy support such as tax reduction can be given appropriately so as to give full play to the exemplary leading role of pilot cities and encourage more cities to focus on sustainable development and improve the efficiency of urban carbon emissions with incentive policies.
2. Emphasis on improving the level of innovation and advanced industry is an important path to improving the efficiency of urban carbon emissions, and the role of low-carbon pilot cities should be maximized from the perspective of improving the level of urban innovation and optimizing the industrial structure of cities. Firstly, it should raise the level of innovation in the city, increase investment in research and innovation, nurture innovative talents in industries related to low-carbon development, attract innovative talents to settle in the city, and provide incentives and an innovative production environment for research and innovation talents. Secondly, it should focus on promoting the advanced industrial structure, enhancing the modernization of the industrial chain, greening the industrial development, promoting the upgrading and optimization of the industrial structure, and promoting the transformation of the industry to low carbon by creating a low carbon industrial development system in the city and establishing low carbon industrial parks.
3. Based on the advantages of regional resource endowments, implement differentiated responses to low-carbon pilot projects according to local conditions. The low-carbon pilot policy has a significant effect on carbon efficiency in the eastern and western regions, in large cities and non-resource-based cities, but not in the central region, in small-sized and medium-sized cities, or in resource-based cities. For regions with significant roles, they should continue to adhere to the development of low-carbon strategies, summarize regional development experience, strengthen cooperation with other regions, help regions with weaker development of low-carbon industries, achieve inter-regional synergistic development, win-win cooperation, and jointly improve the efficiency of carbon emissions. For areas with insignificant effects, they should learn from the experience and methods of areas with significant effects and establish targeted policies suitable for local development so as to narrow the gap in urban carbon emission efficiency and thus ensure the effectiveness of low-carbon pilot policies.
4. Deepen low-carbon pilot work, carry out international exchanges and cooperation, and provide empirical evidence for international low-carbon work. This paper proves that the low-carbon pilot policy can effectively improve the efficiency of urban carbon emissions. As a global carbon emitter, the conclusions drawn by China are of practical significance. In the future, we should focus on the impact of cross-border cooperation on international environmental protection. Internationally, it is recommended to summarize China’s experience, actively carry out low-carbon pilot work in various countries, and encourage more countries to participate in the World Alliance of Low-carbon Cities, so as to achieve the purpose of improving carbon emission efficiency. For China, low-carbon pilot provinces have gradually become a hot spot of international cooperation and an important platform for China’s international exchange and cooperation in addressing climate change. It is recommended to strengthen the international exchange of low-carbon pilot experience, promote the results of low-carbon pilot projects internationally, and learn from the experience of other countries to create a new win-win situation for international low-carbon work.

## Supporting information

S1 Data (XLSX)
